The article "Research on Data Analysis of Traditional Chinese Medicine with Improved Differential Evolution Clustering Algorithm" was published in 2021. Journal: J Healthc Eng.

# Research on Data Analysis of Traditional Chinese Medicine with Improved Differential Evolution Clustering Algorithm

**DOI:** 10.1155/2021/4468741

**Published:** 2021-09-04

**Authors:** Honglei Zhu, Yingying Zhao, Xueyun Wang, Yulong Xu

**Affiliations:** School of Information & Technology Henan University of Chinese Medicine, Zhengzhou 450046, China

## Abstract

Medical data analysis is an important part of intelligent medicine, and clustering analysis is a commonly used method for data analysis of Traditional Chinese Medicine (TCM); however, the classical *K*-Means algorithm is greatly affected by the selection of initial clustering center, which is easy to fall into the local optimal solution. To avoid this problem, an improved differential evolution clustering algorithm is proposed in this paper. The proposed algorithm selects the initial clustering center randomly, optimizes and locates the clustering center in the process of evolution iteration, and improves the mutation mode of differential evolution to enhance the overall optimization ability, so that the clustering effect can reach the global optimization as far as possible. Three University of California, Irvine (UCI), data sets are selected to compare the clustering effect of the classical *K*-Means algorithm, the standard DE-*K*-Means algorithm, the *K*-Means++ algorithm, and the proposed algorithm. The experimental results show that, in terms of global optimization, the proposed algorithm is obviously superior to the other three algorithms, and in terms of convergence speed, the proposed algorithm is better than DE-*K*-Means algorithm. Finally, the proposed algorithm is applied to analyze the drug data of Traditional Chinese Medicine in the treatment of pulmonary diseases, and the analysis results are consistent with the theory of Traditional Chinese Medicine.

## 1. Introduction

Clustering belongs to unsupervised learning, so it can improve the objectivity of the results when applied to medical research. The earliest application of clustering technology to assist medical diagnosis was in the 1970s [1]. With the rapid development of intelligent medicine in 5G era, some scholars study the medical auxiliary diagnosis and have made some achievements [2–5]. For example, Xu et al. simulated the process of TCM diagnosis and created an online analysis platform for TCM based on Latent Tree to assist TCM diagnosis. When using clustering to study TCM syndrome differentiation, it can show obvious objectification and quantification characteristics [6, 7]. Therefore, clustering analysis has become a common data analysis method in TCM diagnosis and treatment and provides an objective method for TCM clinical syndrome differentiation and treatment. However, at present, most studies apply clustering to TCM symptoms and syndromes, while few studies apply clustering to drug analysis [7].

The article "Research on Data Analysis of Traditional Chinese Medicine with Improved Differential Evolution Clustering Algorithm" was published in 2021. Journal: J Healthc Eng.

*K*-Means is a classical clustering algorithm, which has the advantages of simple implementation, fast convergence, and high efficiency. However, in the *K*-means clustering algorithm, it is necessary to determine the number of clusters *K* in advance based on experience and randomly select the initial clustering center. Therefore, the results of cluster analysis are greatly affected by the selection of initial clustering center, outliers, and noise data, which will lead to the unstable results and fall into local optimal solution. It is a feasible idea to determine the initial clustering center and optimize the location by the optimization algorithm. Differential Evolution (DE) is a relatively new stochastic optimization algorithm, which has strong robustness and global optimization capability [8]. At present, although some scholars have introduced global optimization algorithms such as genetic algorithm and ant colony algorithm into *K*-Means clustering algorithm [9, 10], the DE algorithm is more efficient and easier to implement than the above optimization algorithms [11–20].

This paper proposes an improved mutation strategy of DE and optimizes the determination problem of *K*-Means clustering center, which can replace the traditional *K*-Means clustering algorithm to update the clustering center continuously. In this way, it can effectively avoid the *K*-Means algorithm falling into the local optimum. Accordingly, the high-quality initial clustering center can be obtained, and the convergence speed of DE also can be improved. To verify the effectiveness of the proposed algorithm, three UCI datasets are used to compare *K*-Means, DE-*K*-Means, and the proposed algorithm. The experimental results show that the proposed algorithm has better clustering effect.

Finally, the proposed algorithm was used to conduct cluster analysis on the data of TCM drugs in the treatment of diffuse interstitial pulmonary disease, and the method that using TCM to treat the disease and the compatibility rule of drugs are obtained. The contributions of this paper are as follows:

1. An improved DE clustering algorithm is proposed for analyzing the data of Traditional Chinese Medicine
2. Experimental studies are used, using UCI standard datasets to verify the performance of the proposed algorithm

The rest of this paper is organized as follows: Section 2 introduces the relevant theories.  Section 3 presents an improved differential evolution-based *K*-Means clustering algorithm.  Section 4 describes the experiment and evaluation.  Section 5 surveys related works and Section 6 concludes the study.

The article "Research on Data Analysis of Traditional Chinese Medicine with Improved Differential Evolution Clustering Algorithm" was published in 2021. Journal: J Healthc Eng.

## 2. Relevant Theories

The clustering algorithm divides similar data objects into the same class when analyzing data, and its definition can be described as follows: the known set *D* = {*O*_1_, *O*_2_,…, *O*_*n*_}, *O*_*i*_ represents the *i*th object, *i* = {1, 2,…, *n*}, *C*_*t*_ = {*O*_*t*1_, *O*_*t*2_,…, *O*_*tn*_}, *C*_*t*_ ⊆ *D*, *t* = {1, 2,…, *k*}, in the set *C*_*t*_, the first subscript *t* represents the category in the set, and the second subscript represents a data object in the category *t*. If proximity (*O*_*i*_, *O*_*j*_) represents the similarity between objects *O*_*i*_ and *O*_*j*_, then each *C*_*t*_ satisfies the following formula:

(1) $$\begin{array}{c} \cup_{t=1}^{k}C_{t}=D. \end{array}$$

For all the C_*x*_, C_*y*_ ∈ D and C_*x*_ ≠ C_*y,*_ if C_*x*_ ∩ *C*_*y*_ = *ϕ* (only for rigid clustering), then

(2) $$\begin{array}{c} {\text{MIN}}_{\forall O_{xu}O_{xv}\in C_{x,}\forall C_{x}\subseteq D\left(\text{Similarity}\left(O_{xu,}O_{xv\;}\right)\right)}>{\text{MAX}}_{\forall O_{xm}\in C_{x,}O_{yn}\in C_{y,}\forall C_{x}C_{y}\subseteq D\left(\text{Similarity}\left(O_{xm,}O_{yn}\right)\right)}. \end{array}$$

The result of clustering is that the data in the same category are less different from each other and have greater similarity, and the data of different categories have large differences and small similarity. The similarity between the data is estimated based on the property values of the data objects and is measured by density, distance, connectivity, etc. The distance between data objects is taken as the measurement indicators. The smaller the distance, the greater the similarity. Similarly, the larger the distance, the smaller the similarity. At present, a variety of distance calculation formulas are available; the most commonly used are as follows [1].

Manhattan distance:

(3) $$\begin{array}{c} d\left(O_{i},O_{j}\right)=\sum_{k=1}^{n}\left|O_{ik}-O_{jk}\right|. \end{array}$$

Euclidean distance:

(4) $$\begin{array}{c} d\left(O_{i},O_{j}\right)=\sqrt{\sum_{k=1}^{n}{\left(O_{ik}-O_{jk}\right)}^{2}.} \end{array}$$

Cosine distance:

(5) $$\begin{array}{c} d\left(O_{i},O_{j}\right)=\frac{\sum_{1}^{k}\left(O_{ik}\times O_{jk}\right)}{\sqrt{\sum_{1}^{k}O_{ik}^{2}}\times \sqrt{\sum_{1}^{k}O_{jk}^{2}}}. \end{array}$$

The data object *O*_*i*_ = {*O*_*i*1_, *O*_*i*2_,…, *O*_*in*_}, and *n* represents that the data object has *n* attributes.

### 2.1. *K*-Means Algorithm

*K*-Means algorithm belongs to hard clustering algorithm, which is a prototype-based objective function clustering method. It obtains the optimized objective function by calculating the distance from data points to the prototype and obtains the adjustment rules of iterative operation by using the function to calculate the extreme value.

The article "Research on Data Analysis of Traditional Chinese Medicine with Improved Differential Evolution Clustering Algorithm" was published in 2021. Journal: J Healthc Eng.

### 2.2. Differential Evolution Algorithm

Differential Evolution (DE) is a population-based heuristic algorithm, which has the characteristics of strong robustness, high speed, and simple structure. The basic operations of Differential Evolution algorithm include mutation, crossover, selection, and iteration. Its process is briefly introduced below.

First of all, the DE algorithm needs to initialize the parameters and generate the initial population randomly. Then, mutation operations operation is performed on the population. The common mutation strategies are as follows:

DE/rand/1:
  (6) $$\begin{array}{c} v_{i}\left(g\right)=x_{r_{1}}\left(g\right)+F\times \left[x_{r_{2}}\left(g\right)-x_{r_{3}}\left(g\right)\right]. \end{array}$$
DE/best/1:
  (7) $$\begin{array}{c} v_{i}\left(g\right)=x_{\text{best}}\left(g\right)+F\times \left[x_{r_{1}}\left(g\right)-x_{r_{2}}\left(g\right)\right]. \end{array}$$
DE/current-to-best/1:

(8) $$\begin{array}{c} v_{i}\left(g\right)=x_{i}\left(g\right)+F\times \left[x_{\text{best}}\left(g\right)-x_{i}\left(g\right)\right]+F\times \left[x_{r_{1}}\left(g\right)-x_{r_{2}}\left(g\right)\right]. \end{array}$$

After that, the cross operation is performed to improve the diversity of the population, and binomial crossover is generally selected as follows:

(9) $$\begin{array}{c} u_{i,j}\left(g\right)=\left\{\begin{array}{cc} v_{i,j}\left(g\right), & \text{if }{\text{rand}}_{i,j}\left[0,1\right]\leq CR\text{ or }j=j_{\text{rand}},\\ x_{i,j}\left(g\right), & \text{ otherwise.} \end{array}\right) \end{array}$$

Binomial crossover intersects the generated mutation vector *V*_*i*_(*g*) with the parent individual vector *X*_*i*_(*g*) to obtain the experimental vector *U*_*i*,*j*_(*g*), in which the symbol *U*_*i*,*j*_(*g*) represents the *j*th gene of the *i*th individual in the *g* generation populations, *j* = 1, 2,…, *D*, and *D* denotes the dimension of the problem. The symbol *j*_rand_ denotes a random integer with uniform distribution in [1, *D*], which ensures that at least one dimension of the experimental vector comes from the mutation vector. Crossover probability CR controls the convergence speed of the algorithm, and CR ∈ [0, 1].

Finally, the selection operation is performed, in which the excellent individuals with the optimal objective function value are preserved and evolved into the next generation. Take the solution minimization as an example, as shown in the following equation:

(10) $$\begin{array}{c} x_{i}\left(g+1\right)=\left\{\begin{array}{cc} u_{i}\left(g\right), & \text{if }f\left(u_{i}\left(g\right)\right),\\ x_{i}\left(g\right), & \text{ otherwise.} \end{array}\right) \end{array}$$

The article "Research on Data Analysis of Traditional Chinese Medicine with Improved Differential Evolution Clustering Algorithm" was published in 2021. Journal: J Healthc Eng.

## 3. Improved Differential Evolution-Based *K*-Means Clustering Algorithm

### 3.1. Population Initialization

The clustering algorithm based on DE randomly generates the initial population POP = [*x*_1_, *x*_2_, *x*_3_,…, *x*_*NP*_], *x*_*i*_ = [*x*_*i,*1_, *x*_*i,*2_, *x*_*i,*3_,…, *x*_*i,D*_]; the symbols *NP* and *D* denote the population size and the data dimension, respectively. Compared with the traditional *K*-Means algorithm, it can provide a larger search space for finding the optimal clustering center.

### 3.2. Population Diversity-Based Double-Mutation Operation

#### 3.2.1. Population Diversity Calculation

The ability of the algorithm to search the optimal solution depends on the current population diversity. Tang et al. [21] defined the population similarity coefficient to judge the population diversity, and Wang et al. [22] defined the variance of the population fitness value to reflect the aggregation degree of all individuals in the population. Referring to their studies, this paper proposes a new indicator *λ*_(*g*)_ to evaluate population diversity, and the indicator *λ*_(*g*)_ can be calculated by the following formulas:

(11) $$\begin{array}{c} \mu_{\left(g\right)}=\frac{1}{\text{NP}}\sum_{i=1}^{\text{NP}}x_{i}\left(g\right), \end{array}$$

(12) $$\begin{array}{c} \sigma_{\left(g\right)}=\sqrt{\frac{1}{\text{NP}}\sum_{i=1}^{\text{NP}}{\left(x_{i}\left(g\right)-\mu_{\left(g\right)}\right)}^{2}}. \end{array}$$

(13) $$\begin{array}{c} \lambda_{\left(g\right)}=\frac{\sigma_{\left(g\right)}}{\mu_{\left(g\right)}}. \end{array}$$

Here, the symbols NP, *x*_*i*_(*g*), *μ*(*g*), and *σ*(*g*) represent the population size, the individual *i* of *g*th generation, the central individual in the population, and the average distance from all individuals in the population to the central individual. As shown in Figure 1, it is assumed that there are three individuals *x*_1_, *x*_2_, and *x*_3_ in the population, and the central individual is *μ*(*g*). The larger the value of *λ*(*g*), the greater the distance between individuals, that is, the better the diversity. The smaller the value of *λ*(*g*), the worse the population diversity, and the individuals in the population are more clustered.

#### 3.2.2. Double-Mutation Strategy

In the evolution process, in order to balance the development ability and convergence speed of algorithm, Zhang and Sanderson [23] and Islam et al. [24] adopted a new mutation strategy, and Qin et al. [25] and Yi et al. [26] proposed the multimutation strategy. Based on the previous studies, this paper combines two mutation strategies to carry out mutation operation on individual population, which is recorded as double-mutation operation. That is, according to the current population diversity, the appropriate mutation strategy is selected.

(14) $$\begin{array}{c} v_{i}\left(g\right)=\left\{\begin{array}{cc} x_{r_{1}}\left(g\right)+F\times \left[x_{r_{2}}\left(g\right)-x_{r_{3}}\left(g\right)\right],\; & \lambda_{\left(g\right)}<\text{Threshold,}\\ x_{\text{best}}\left(g\right)+F\times \left[x_{r_{1}}\left(g\right)-x_{r_{2}}\left(g\right)\right], & \text{otherwise.} \end{array}\right) \end{array}$$

As shown in formula (14), in the early stage of evolution, the population diversity is good, and the value of *λ*(*g*) is greater than the set threshold. At this time, the mutation strategy DE/best/1 is selected to guide the search direction of the population with the optimal individual, which can enhance the development ability of the algorithm and accelerate the convergence speed of the algorithm. With the increase of evolution generation, the population diversity will rapidly decline. When the population diversity evaluation indicator is less than the set threshold, the mutation strategy DE/rand/1 is selected, which selects individuals randomly to guide the search direction and improves the population diversity to avoid falling into the local optimal solution.

The article "Research on Data Analysis of Traditional Chinese Medicine with Improved Differential Evolution Clustering Algorithm" was published in 2021. Journal: J Healthc Eng.

In evolution algorithms, population diversity is generally approximate to the variance of individual variable values. The larger the variance, the higher the diversity. The average indicator *λ*(*g*) proposed in this paper includes the distance from all individuals to the central individual, which belongs to the variation of variance measurement and can reflect the change of population diversity.

### 3.3. Fitness Function

Clustering belongs to unsupervised learning method. When using evolution algorithm to solve the clustering, it should be transformed into an optimization problem at first, and the optimal objective function (i.e., fitness function) should be established. In this paper, the sum of within-class distances (WCD) is taken as the fitness function.

(15) $$\begin{array}{c} \text{wcd}=\sum_{k=1}^{k}\sum_{i=1}^{m_{k}}x_{i}^{k}-c_{k}. \end{array}$$

As shown in formula (15), the symbols *k*, *m*_*k*_, *x*_*i*_^*k*^, and *c*_*k*_ represent the number of clustering, the total number of data in the *K* class, the *i*th data in the *K* class, and the clustering center of the *K* class, respectively. In this paper, formula (4) is used to calculate the distance from each data point to each clustering center. The smaller the value of WCD, the more concentrated the data points in various types, and the better the clustering effect; that is, the minimization of WCD is solved.

The article "Research on Data Analysis of Traditional Chinese Medicine with Improved Differential Evolution Clustering Algorithm" was published in 2021. Journal: J Healthc Eng.

### 3.4. Improved Differential Evolution Clustering Algorithm

The improved DE is combined with *K*-Means clustering algorithm to obtain the optimized clustering algorithm, that is, the clustering algorithm based on the improved differential evolution. The initial clustering center of the algorithm is randomly selected, and the optimal location of the clustering center is realized in the evolution process, so that the final clustering result can reach the global optimal. The overall flow of the algorithm is given in Algorithm 1.

In Algorithm 1, the population POP and each parameter value should be initialized at first. Then, according to formula (15), the objective function value of each individual can be calculated, and the current optimal value can be obtained. After that, the indicator of population diversity is calculated by formulas (11)–(13), and the mutated individual is obtained by directing all individuals to perform variation operations based on current population diversity. Then, the experimental individuals can be obtained by performing cross operation on the mutated individuals. Formula (15) is used to evaluate the fitness of experimental individuals and contemporary individuals, and the better individuals are selected to enter the next generation; accordingly, the objective function value of the optimal individual is retained. Finally, the algorithm will go to statement 3 for execution until the optimal solution is obtained or the maximum number of iterations is reached.

## 4. Simulation Experiment and Analysis

### 4.1. UCI Standard Test Set

In order to verify the performance of the algorithm, this paper compares *K*-Means, *K*-Means++, and DE-*K*-Means clustering algorithm with the proposed algorithm. Three data sets were selected from the UCI as test datasets, and the properties are described in Table 1.

In the DE-*K*-Means algorithm and the proposed algorithm, the mutation factor *F* is set to 0.6, the crossover probability CR is set to 0.5, the population size *NP*=10^*∗*^ dim, and the threshold value of *λ* in the proposed algorithm is set to 0.005. Moreover, dim represents the number of individual attributes. If the algorithm converges to the same optimal solution more than 400, then the algorithm is terminated. The maximum evaluation times is 1500, and each algorithm will run 40 times independently for the test set. The simulation software used in the experiment is MATLAB R2016b.

The clustering results are shown in Tables 2–4, the maximum value, minimum value, and average value of the inner-class distance which are obtained through 40 independent experiments on three UCI datasets. From these experimental results, it can be seen that *K*-Means algorithm and *K*-Means++ algorithm have a fast convergence speed with the least number of iterations. However, there is a large gap between the maximum and minimum values of the inner-class distance, and the results fluctuate greatly. Moreover, the tightness between data in the same class is poor, and the stability of clustering results needs to be improved. Compared with *K*-Means and *K*-Means++ algorithms, the objective function value optimized by DE-*K*-Means algorithm and the proposed algorithm are better, the stability and accuracy of clustering results are improved, and the clustering results obtained by the proposed algorithm are better. In short, the performance of the proposed algorithm is better than other algorithms in three datasets, especially in the Zoo dataset.

The article "Research on Data Analysis of Traditional Chinese Medicine with Improved Differential Evolution Clustering Algorithm" was published in 2021. Journal: J Healthc Eng.

The comparisons of convergence curves between DE-*K*-Means algorithm and the proposed algorithm on UCI data are shown in Figures 2–4. It is found that, compared with DE-*K*-Means algorithm, the target function value of the proposed algorithm tends to be optimal earlier; that is, the convergence speed of the proposed algorithm is better than that of the DE-*K*-Means algorithm. To sum up, the proposed algorithm performs well in stability, accuracy, and convergence speed.

### 4.2. Data Comparison of Lung Diseases in Traditional Chinese Medicine

Diffuse pulmonary interstitial disease is characterized by alveolar damage and interstitial fibrosis [27]. Since it has high morbidity and mortality, with the deterioration of air quality, how to prevent the disease and the usage of drugs for disease are the hot spots that people pay attention to. In this paper, the clustering algorithm based on differential evolution is used to analyze the usage rules of prescriptions of Traditional Chinese Medicine in the treatment of diffuse interstitial lung disease.

The data of this section comes from the “Database of Literature Research on the Diagnosis and Treatment of Diffuse Pulmonary Interstitial Disease by modern famous veteran doctors of TCM,” which contains 39 kinds of TCM works and 16 literatures, with a total of 270 data [28].

Based on the experimental results of the UCI dataset, in this section, the DE-*K*-Means algorithm and the proposed algorithm are used for clustering the drug data of diffuse interstitial pulmonary disease (hereinafter referred to as TCM data). In these two algorithms, the values of variation factor *F* and crossover probability CR are set to 0.6 and 0.5, respectively, and the population size NP equals 10∗dim. The threshold value *λ* in the proposed algorithm is set to 0.001. If the algorithm converges to the same optimal solution more than 400 times, the algorithm will be terminated. The maximum number of evaluations is 2500. Each algorithm will independently run the data for 40 times. The simulation software used in experiments is MATLAB R2016b.

The article "Research on Data Analysis of Traditional Chinese Medicine with Improved Differential Evolution Clustering Algorithm" was published in 2021. Journal: J Healthc Eng.

A reasonable experience value *K* = 7 can be obtained by analyzing and comparing the experimental results of the number of different categories. The experimental clustering results are shown in Table 5. The convergence graphs of DE-*K*-Means and the proposed algorithm on the given data are shown in Figures 5 and 6, respectively.

From Table 5 and Figures 5 and 6, it can be seen that the clustering effect of the proposed algorithm is better than the DE-*K*-Means algorithm for TCM data. Combined with the theory of TCM, the seven clustering results are described as follows.

The main drugs of class 1 include *Angelica*, *Astragalus membranaceus*, honeysuckle, and raw *Astragalus*. Among them, *Astragalus membranaceus* can nourish the middle and Qi. *Angelica* can replenish blood and activate blood. Honeysuckle can clear away heat and detoxify. Raw *Astragalus* can nourish the surface and stop sweating and invigorate the Qi and Yang. These drugs are matched to replenish Qi and blood, replenish diarrhea, and clear away heat and toxins. It is applicable to those who have the syndrome of deficiency of Qi and Yin, deficiency of Qi and blood, and stagnation of heat and toxin.

The main drugs of class 2 include *Salvia miltiorrhiza*, *Angelica sinensis*, red peony root, and *Ligusticum wallichii*. Among them, *Salvia miltiorrhiza* can activate blood circulation and regulate menstruation and can cool blood to eliminate carbuncle. Red peony root can clear heat and cool blood and can activate blood circulation to remove blood stasis. *Ligusticum wallichii* can open depression and can activate blood and relieve pain. These drugs are matched to promote blood circulation and remove blood stasis and are suitable for the symptoms caused by blood stasis.

The main drugs of class 3 include *Fritillaria sichuanensis*, *Fritillaria thunbergii*, *Scutellaria baicalensis* Georgi, and *Schisandra chinensis*. Among them, *Fritillaria sichuanensis* can clear away heat and moisten the lung, dissipate phlegm and stop cough, and can disperse the knot and eliminate carbuncle. *Fritillaria thunbergii* can clear away heat and phlegm and stop cough, detoxify the knot, and eliminate carbuncle. *Scutellaria baicalensis* can clear away heat and dry dampness and can relieve fire and detoxify. *Schisandra chinensis* can collect lung and stop cough and can nourish astringent essence. The combination of these drugs can clear the heat and reduce phlegm, which is suitable for the syndrome of phlegm-heat accumulated in lung.

The article "Research on Data Analysis of Traditional Chinese Medicine with Improved Differential Evolution Clustering Algorithm" was published in 2021. Journal: J Healthc Eng.

The main drugs of class 4 include *Ophiopogon japonicus*, *Adenophora verticillata*, *Schisandra chinensis*, *Fritillaria sichuanensis*, almond, coix seed, Flos Farfarae, cortex mori, and aster. Among them, *Ophiopogon japonicus* can promote the secretion of saliva to quench thirst and can moisten lung to stop coughing. *Adenophora verticillata* can nourish yin and clear heat, moisten lung and dissipate phlegm, benefit stomach, and generate body fluid. Almond can relieve cough and asthma, moisten intestines, and relieve constipation. Coix seed can invigorate the spleen to arrest diarrhea, clear damp, and promote diuresis. Flos Farfarae can relieve cough. Aster can dissipate phlegm. Cortex Mori can purge the lung to calm panting, and induce diuresis to alleviate edema. The combination of these drugs can dissolve phlegm and arrest cough, moistening lung and promoting fluid production, which are suitable for the syndrome cough and asthma with deficiency of Qi and Yin and stagnation of phlegm heat.

The main drugs of class 5 include *Codonopsis pilosula* and licorice. Among them, *Codonopsis pilosula* can tonify middle-Jiao and Qi, strengthen spleen, and tonify lung. Licorice can tonify spleen and Qi, expel phlegm to arrest coughing, and relieve spasm and pain. The combination of these two drugs can invigorate the spleen and lung, which are suitable for the syndrome of deficiency of lung and spleen.

The main drugs of class 6 include honeysuckle, *Trichosanthes*, loquat leaf, and licorice. Among them, *Trichosanthes* can clear heat and remove phlegm and moisturize and smooth the intestines; loquat leaf can clear the lungs and relieve cough. These drugs are matched to clear the heat and reduce phlegm, and it is suitable for the wind heat to make the lung cough and asthma on the inverse.

The main drugs of class 7 include tuckahoe and atractylodes. Among them, tuckahoe can clear damp and promote diuresis and tonify spleen and heart. Atractylodes can tonify the spleen and strengthen the stomach. These two drugs are matched to strengthen the spleen and dampness, which is suitable for the syndrome of deficiency of spleen.

The analysis of the above seven clustering results is consistent with the basic knowledge of Traditional Chinese Medicine. In the treatment of diffuse pulmonary interstitial disease, there are both clearing heat, resolving phlegm, relieving cough, relieving asthma, promoting blood circulation, removing blood stasis, eliminating dampness and clearing damp and tonifying Qi, nourishing Yin, enriching blood, vitality, profiting lung, tonifying the spleen and kidney, so as to support the main etiology and pathogenesis of diffuse pulmonary interstitial disease is the combination of deficiency and excess.

The article "Research on Data Analysis of Traditional Chinese Medicine with Improved Differential Evolution Clustering Algorithm" was published in 2021. Journal: J Healthc Eng.

## 5. Related Works

Differential evolution has emerged as one of the fast, robust, and efficient global search heuristics of current interest. Das et al. [11] described an application of DE to the automatic clustering of large unlabeled data sets. In contrast to most of the existing clustering techniques, the proposed algorithm requires no prior knowledge of the data to be classified. To study whether the performance of DE can be improved by combining several effective trial vector generation strategies with some suitable control parameter settings, Wang et al. [12] proposed a novel method, called composite DE (CoDE), which uses three trial vector generation strategies and three control parameter settings and randomly combines them to generate trial vectors. For the unconstrained global optimization problems, Liu et al. [13] proposed a hybrid DE based on the one-step *k*-means clustering and 2 multiparent crossovers, called clustering-based differential evolution with 2 multiparent crossovers (2-MPCs-CDE). In their method, the *k* cluster centers and several new individuals generate two search spaces. Xu et al. [14] proposed a superior-inferior (SI) crossover scheme based on DE. In their scheme, when population diversity degree is small, the SI crossover is performed to improve the search space of population. Otherwise, the superior-superior crossover is used to enhance its exploitation ability. Mohamed et al. [15, 16] proposed an adaptive guided differential evolution algorithm (AGDE) for solving global numerical optimization problems over continuous space, and they also propose a novel differential evolution algorithm, called NDE, for solving constrained engineering optimization problems. The key idea of the proposed NDE is the use of new triangular mutation rule, which is used to search for better balance between the global exploration ability and the local exploitation tendency as well as enhancing the convergence rate of the algorithm through the optimization process. Meng et al. [18, 19] proposed the parameter adaptive DE (PaDE) to tackle the weaknesses of DE, such as the improper control parameter adaptation schemes and the defect in a given mutation strategy. They also proposed a novel DE variant, named Depth information-based Differential Evolution with adaptive parameter control for numerical optimization (Di-DE), in which the novel mutation strategy, grouping strategy, and cooperative strategy are adopted to tackle the weaknesses of DE, such as the premature convergence to some local optima of a mutation strategy and the misleading interaction among control parameters. Wang et al. proposed a self-adaptive mutation differential evolution algorithm based on particle swarm optimization (DEPSO) to improve the optimization performance of DE, in which the population diversity can be maintained well in the early stage of the evolution, and the faster convergence speed can be obtained in the later stage of the evolution.

The article "Research on Data Analysis of Traditional Chinese Medicine with Improved Differential Evolution Clustering Algorithm" was published in 2021. Journal: J Healthc Eng.

## 6. Conclusions

This paper proposes an improved differential evolution algorithm, which uses a new indicator to evaluate population diversity, and adopts the double-mutation strategy according to the current population diversity. The improved DE is applied to *K*-Means clustering to optimize and locate the clustering center, which can improve the performance and stability of clustering algorithm. The simulation results show that the improved clustering algorithm can improve the global optimization and convergence speed. Finally, the improved clustering algorithm is used to analyze the medication data of TCM in the treatment of pulmonary diseases. The clustering results are in accord with the theory of Traditional Chinese Medicine, which verify that the main etiology and pathogenesis of pulmonary diseases are intermingled deficiency and excess, deficient root and excessively superficial. As a whole, it not only provides reference for clinical treatment, but also verifies the practicability of the proposed method.

## Figures and Tables

**Figure 1:** The central individual *μ*(*g*).

**Figure 2:** The standard DE-*K*-Means Iris convergence curve (a) and the improved DE-*K*-Means Iris convergence curve (b).

**Figure 3:** The standard DE-*K*-Means Wine convergence curve (a) and the improved DE-*K*-Means Wine convergence curve (b).

**Figure 4:** The standard DE-*K*-Means Zoo convergence curve (a) and the improved DE-*K*-Means Zoo convergence curve (b).

**Figure 5:** The convergence curve of DE-*K*-Means algorithm.

**Figure 6:** The convergence curve of the proposed algorithm.

**Algorithm 1:** Improved differential evolution clustering algorithm.

**Table 1:** The base information of datasets.

Datasets	Number of data	Number of attributes	Number of classes
Iris	150	4	3
Wine	178	13	3
Zoo	101	16	7

**Table 2:** The clustering results of Iris.

Algorithm	Minimum inner-class distance	Maximum inner-class distance	Mean inner-class distance	Mean number of iterations
*K*-Means	97.3259	123.8497	103.042985	7.1
*K*-Means++	97.3259	122.4787	100.461185	6.6
DE-*K*-Means	96.6555	97.3365	96.6725675	1109.3
Proposed	96.6555	96.6555	96.6555	549.8

**Table 3:** The clustering results of Wine.

Algorithm	Minimum inner-class distance	Maximum inner-class distance	Mean inner-class distance	Mean number of iterations
*K*-Means	16555.6794	18436.9521	16953.75104	7.9
*K*-Means++	16555.6794	18436.9521	17384.2979	8.0
DE-*K*-Means	16292.1846	16295.1591	16292.43106	1500.0
Proposed	16292.1846	16292.6672	16292.19667	1319.2

The article "Research on Data Analysis of Traditional Chinese Medicine with Improved Differential Evolution Clustering Algorithm" was published in 2021. Journal: J Healthc Eng.

**Table 4:** The clustering results of Zoo.

Algorithm	Minimum inner-class distance	Maximum inner-class distance	Mean inner-class distance	Mean number of iterations
*K*-Means	101.9719	133.4409	110.77463	5.0
*K*-Means++	101.9719	118.4956	109.392745	3.9
DE-*K*-Means	101.3131	126.2266	106.9885275	1500.0
Proposed	101.1552	107.9804	104.4135725	1500.0

**Table 5:** The clustering results of TCM data.

Algorithm	Minimum inner-class distance	Maximum inner-class distance	Mean inner-class distance
DE-*K*-Means	493.9222	524.8227	501.462525
Proposed	489.2295	507.5878	496.5335875

## Data Availability

The data used to support the findings of this study are available from the corresponding author upon request.
